# High Glucose Promotes Pancreatic Ductal Adenocarcinoma Gemcitabine Resistance and Invasion through Modulating ROS/MMP-3 Signaling Pathway

**DOI:** 10.1155/2022/3243647

**Published:** 2022-09-29

**Authors:** Junyuan Deng, Yujie Guo, Xiaomu Hu, Jiali Du, Jichun Gu, Lei Kong, Baian Tao, Deliang Fu, Tianlei Ying, Ji Li

**Affiliations:** ^1^Department of Pancreatic Surgery, Pancreatic Disease Institute, Huashan Hospital, Fudan University, 12 Wulumuqi Middle Road, Shanghai 200040, China; ^2^Department of Pathology, Huashan Hospital, Fudan University, Shanghai 200040, China; ^3^MOE/NHC/CAMS Key Laboratory of Medical Molecular Virology, School of Basic Medical Sciences, Fudan University, Shanghai 200032, China

## Abstract

Pancreatic ductal adenocarcinoma (PDA) is often concomitant with diabetes mellitus, which mainly manifests as an increased blood glucose level. Previous studies revealed that diabetic status reduced the survival and blunted gemcitabine sensitivity in PDA patients. This study is aimed at analyzing the mechanism of elevated gemcitabine resistance and cancer invasion ability under high glucose environment. We selected 129 patients with 22 surgical resected samples from 2015 to 2021, who underwent pancreatic surgery in Huashan Hospital. The gene expression and clinical data of PDA were obtained from The Cancer Genome Atlas (TCGA) website and were analyzed by R software. Cell viability assays and flow cytometry were applied to detect gemcitabine sensitivity and apoptosis levels in pancreatic cancer cells. Wound healing and Transwell tests were used to analyze the invasion and metastasis of cancer cells. Streptozotocin (STZ) was used to establish a hyperglycemic mouse model for the *in vivo* study. In this study, diabetic PDA gemcitabine users showed reduced survival compared to euglycemic PDA gemcitabine users. Clinical samples and laboratory studies revealed that MMP-3 expression was associated with glucose concentration and diabetic status. Elevated MMP-3 expression was positively related to cancer invasion and gemcitabine resistance in PDA cells and gemcitabine resistant PDA cells. Blocking MMP-3 expression inhibited gemcitabine resistance and cancer progression in cellular and animal models. MMP-3 was closely related to the expression of RRM1, a gemcitabine metabolism-related gene. Reactive oxygen species (ROS) level increased under higher glucose concentrations and was mediated by NOX4. ROS determined the MMP-3 expression in pancreatic cancer cells. Inhibiting NOX4 expression effectively suppressed MMP-3 expression, gemcitabine resistance, and cancer invasion. In conclusion, a high glucose environment induces gemcitabine resistance and cancer invasion via ROS/MMP-3 signaling pathway. MMP-3 can be a potential novel target for suppressing gemcitabine resistance and invasion in PDA.

## 1. Introduction

Pancreatic ductal adenocarcinoma (PDA), often referred to as pancreatic cancer, is a devastating disease that ranks the fourth leading cause of cancer-related death and is projected to be the second leading cause of death by 2030 in the United States [1]. Currently, the 5-year survival of PDA patients is lower than 10%, and over 80% of cases were unresectable when diagnosed. Currently, chemotherapy is a crucial method for prolonging PDA patients' survival. Gemcitabine (GEM), a nucleoside analog of deoxycytidine, inhibits pancreatic cancer through interfering DNA synthesis. After being treated with gemcitabine, increased cell apoptosis and decreased cell viability were observed in pancreatic cancer cells. Since its approval by the FDA in 1996, gemcitabine has been extensively used to treat various solid tumors and currently in certain lymphomas [2, 3]. At present, as no alternative therapeutic options exist, gemcitabine is vital for neoadjuvant, adjuvant, and palliative therapy in PDA. However, the problem is that the relatively low gemcitabine response rate (less than <30%) is consistently disturbing PDA patients [4].As a chronic disease, diabetes mellitus (DM) is often concomitant with PDA. Epidemiological evidence revealed that over 50% of PDA patients had DM, and over 75% of PDA cases reported were hyperglycemia. Unlike typical type 2 diabetes mellitus (T2DM), diabetes in PDA patients manifests as hyperglycemia with normal or relatively lower insulin levels caused by the removal of normal pancreatic tissue. Aside from this, diabetic patients showed a significant reduction in overall survival compared with euglycemic patients, especially those who received gemcitabine-based chemotherapy. Currently, the mechanism of how high glucose initiates tumorigenesis and PDA development is well studied. However, unfortunately, a systematic understanding of how diabetes interferes with gemcitabine sensitivity in pancreatic cancer is still not clear at present.

This study is aimed at clarifying the potential mechanism of how high glucose induces gemcitabine resistance and metastasis in pancreatic cancer. And we also delivered a novel target for suppressing PDA progression and chemoresistance induced by hyperglycemia.

## 2. Materials and Methods

### 2.1. Public Database Data Download

The Cancer Genome Atlas (TCGA), sponsored by National Cancer Institute, is a publicly available database containing multidimensional cancer genomics and clinical data sets. We downloaded pancreatic adenocarcinoma (PAAD) clinical information and RNA sequence data from the Broad Firehose Website (http://gdac.broadinstitute.org). In the TCGA-PAAD cohort, patients that had a history of diabetes were regarded as having pancreatic cancer with diabetes (the diabetic cohort). In contrast, pancreatic cancer individuals without a history of diabetes were considered as PAAD without diabetes (the normal cohort). Cases with no clear diabetes history were excluded from our study. The RNA sequence data of GSE50931 was downloaded from the GEO (Gene Expression Omnibus) database to evaluate the downstream effectors of MMP-3 involved in PDA gemcitabine resistance.

### 2.2. Identification of Differentially Expressed Genes (DEGs)

The DEGs analysis was performed on two categories of samples according to the diabetes history (the normal cohort and the diabetic cohort) or the MMP-3 expression (the high MMMP-3 expression cohort and the low MMP-3 expression cohort). Limma R package was used to identify the differentially expressed genes between the normal and diabetic cohorts, which were defined as those with a false discovery rate <0.05 and a |fold change| > 1. The heat map analysis of the mRNA expression pattern was performed using R software with the “edgeR” package.

### 2.3. Univariate Cox Analysis and LASSO Regression Analysis

We applied survival-related univariate Cox analysis and LASSO regression analysis to determine the critical factor in PDA patients' survival. After eliminating the patient data with no survival time, the DEGs with positive prognosis in the TCGA cohort were determined by univariate Cox analysis. After screening the DEGs with survival univariate Cox analysis, LASSO regression analysis was performed to examine the key factors furtherly. The algorithm of LASSO regression was conducted with the Glmnet R package to select and shrink variables by excluding the variables with a regression coefficient equal to 0. Then, an interpretable model was established according to the nonzero regression coefficients in the TCGA cohort, and the optimum *λ* was selected in 10-fold cross-validation. We calculated the risk scores of each DEGs and its corresponding regression coefficient based on risk scores in the TCGA cohort.

### 2.4. ROC Model Construction

A time-dependent ROC analysis (1 year, 3 years, and 5 years) was conducted to measure the MMP-3 survival prediction effect using the survival and time ROC R package to assess the prediction accuracy. The sequence data and clinical information were obtained from the TCGA database. Areas under the curve (AUC) were used to measure the survival predicting the efficacy of the prognostic model of MMP-3.

### 2.5. Functional Enrichment Analysis

Functional enrichment analysis, including Gene Set Enrichment Analysis (GSEA), Gene Ontology (GO), and Kyoto Encyclopedia of Genes and Genomes (KEGG) analyses, were used to identify gene sets and pathways correlated with diabetic cohort and high MMP-3 expression cohort. The GSEA software was downloaded from the Broad Institute Website (http://software.broadinstitute.org/gsea/index.jsp), and GSEA analysis was performed according to the manufacturer's instructions. The GO and KEGG analyses based on DEGs were conducted by “clusterProfiler” in R software.

### 2.6. Case Selection and Diabetes Evaluation

The study protocol was authorized by the Ethics Committee of Huashan Hospital, Fudan University. Officially written informed consent was acquired from all patients involved in this study. We strictly selected 129 patients who underwent surgical resection from October 2015 to December 2021, in a high-volume pancreatic center, and all of them had a clear diabetes history or nondiabetic diagnosis. The assessment of diabetes was based on American Diabetes Association (ADA) guidelines and clinical records. The major criteria of DM diagnosis were preoperative fasting plasma glucose ≥12.6 mg/dL, random plasma glucose ≥200 mg/dL, or hemoglobin A1c (HbA1c) ≥6.5%. Patients who had a DM history were also concluded in the DM group [5]. Pancreatic surgery was performed based on malignant signs and patients' decisions. Two independent pathologists made pathological stage evaluations from Huashan Hospital, Fudan University.

### 2.7. Cell Culture

The pancreatic cancer cell lines, BxPc-3, PANC-1, PANC-2, HPDE6-C7, and MiaPaCa-2, were obtained from the National Collection of Authenticated Cell Culture Bank (Shanghai, China). The gemcitabine-resistant BxPc-3 cell line (BxPc-3(GemR)) and its normal control (BxPc-3(Normal)) were obtained from YBR Bioscience, Shanghai, China. All cancer cells were cultured in a DMEM medium containing 10% fetal bovine serum with 1% 100 U/mL penicillin/streptomycin mixture (Beyotime, Shanghai, China). All pancreatic cancer cells were cultured at 37°C with 5% CO_2_. The glucose concentration was 25 mM for normal cell culture, and to evaluate the influence of different glucose environments, two relatively lower glucose concentration levels (5 mM and 15 mM) were created. In this study, 5 mM, 15 mM, and 25 mM glucose concentration group was defined as the Low Glucose Group (LG), Medium Glucose Group (MG), and High Glucose Group (HG), respectively.

### 2.8. Cell Viability Assay

The cells in each group (1 × 10^4^ cells/well) were cultured in 96-well plates with different agents for different times (24 h and 48 h). At each time point, 10 *μ*L of Cell Counting Kit-8 (CCK-8) solution (Beyotime, Shanghai, China) was supplemented into each well and incubated for 1.5 h. Next, the absorbance of each well at 450 nm (OD450 value) was measured by a microplate reader (BioRad Laboratories, Inc., Hercules, CA, United States). The proliferative rate (PR) was measured by: PR = OD450 value (treated group)/OD450 value (normal control group). To adjust the influence of proliferative advantages by high glucose concentration, the normal control groups of HG, MG, and LG were cultured in different glucose levels DMEM.

### 2.9. Western Blotting Assay

After 3 times of PBS washing, all cell lysates were extracted with RIPA lysis buffer (Beyotime, Shanghai, China). 15 *μ*L of each sample was used for SDS-PAGE electrophoresis and transferred to PVDF membranes (Millipore, Billerica, MA, USA). The membranes were blocked in 5% nonfat milk for 1 h and incubated with primary antibody at 4°C overnight. After washing the samples with PBST (fifteen  min/time) three times, the membranes were incubated with a second antibody at room temperature for 1.5 h. After washing three times with PBST, they were visualized with enhanced chemiluminescence (Tanon 3500R, China).

### 2.10. ROS Measurement Assay

ROS assay was purchased from Beyotime, Shanghai, China (S0033S). Intracellular ROS was detected employing an oxidation-sensitive fluorescent probe (DCFH-DA). After being treated with different glucose concentrations DMEM for 24 h, cancer cells were washed three times in phosphate-buffered saline (PBS). They were then incubated with 10 *μ*mol/L DCFH-DA at 37°C for 20 min according to the manufacturer's instructions. DCFH-DA was deacetylated intracellularly by nonspecific esterase, which ROS further oxidized to the fluorescent compound 2,7-dichlorofluorescein (DCF). DCF fluorescence was detected by a microplate reader (BioRad Laboratories, Inc., Hercules, CA, United States).

### 2.11. Transient Transfection Assay

Transient transfection was applied to construct the MMP-3 overexpression cell model and MMP-3 silencing pancreatic cell model. MMP-3 overexpression cDNA (MMP3-GFP-Puro) vector and empty vector cDNA (GAPDH-NC) were designed and synthesized by Mohan (Shanghai, China). The MMP3 siRNAs used for inhibiting MMP-3 expression were designed and synthesized by Ribobio (Guangzhou, China). Lipofectamine™2000 (Invitrogen, California, U.S.A.) was used in the transient transfection process of cDNA and the siRNAs according to the manufacturer's protocol. After transfecting for 16 h, the medium was replaced with 10% FBS High Glucose DMEM, and the transfected cell lines were used for further research.

### 2.12. Apoptosis Detection (Flow Cytometry Assay)

Cell apoptosis and necrosis were determined by Annexin V-FITC/PI double staining and quantified by flow cytometry. Briefly, 1 × 10^6^ cells were harvested and resuspended in 500 *μ*L binding buffer containing 10 *μ*L Annexin V-FITC and 5 *μ*L PI from the Annexin V-FITC/PI Apoptosis Detection Kit (Yeasen, Shanghai, China) for 30 min at room temperature in the dark environment. Then the samples were analyzed using FACSCalibur (BD Biosciences). The living cells were disseminated in Annexin V-FITC−/PI− area (lower left quadrant), early apoptotic cells in Annexin V-FITC+/PI− area (upper left quadrant), late-stage apoptotic cells in Annexin V-FITC+/PI+ area (upper right quadrant), and necrotic cells as Annexin V-FITC−/PI+ (upper left quadrant). Annexin V-FITC/PI Apoptosis Detection Kit was purchased from the Yeasen Corporation, Shanghai, China.

### 2.13. Cell Migration and Invasion Assays

Wound healing and Transwell assays were performed to assess the cell migration and invasion in PDA cells. For wound healing assay, 6-well plates were seeded with 5 × 10^5^ cells and incubated in a humidified atmosphere of 37°C. Until 100% confluence was reached, the layer of cells was scratched with a 100 *μ*L pipette tip (sigma) and washed by PBS three times. Cells were then incubated in fresh serum-free DMEM for an additional 12 hours. The wound closure extent was measured by microscopy. For the Transwell invasion assay, the upper chamber inserts were precoated with 50 *μ*L Matrigel (1 : 4 ratio in high glucose DMEM without FBS) and 3 × 10^3^ cells in 100 *μ*L of serum-free medium were seeded into the upper chamber of each well. Each lower chamber was filled with 600 *μ*L DMEM supplemented with 10% FBS. After 24 h, pancreatic cancer cells were fixed, stained with 500 *μ*L, 4% paraformaldehyde, and 1% crystal violet (Beyotime, Shanghai), respectively. Next, ImageJ software was used to evaluate the number of invasion cells of the corresponding group, and the average of those fields was utilized as a result.

### 2.14. Immunohistochemistry (IHC) Assay and Measurement

Written informed consent of the sample usage was acquired from all patients involved in this study. 22 surgical resected pancreatic cancer samples subjected to antigen were retrieved through incubation in EDTA antigen retrieval buffer (pH 9.0) for 15 min at 100°C. Endogenous peroxidase was blocked by incubation with 3% H_2_O_2_ for 25 min, followed by washes in PBS solution for 5 minutes/3 times. Incubation with 3% bovine serum albumin (BSA) was performed to block other antigens. Incubation with the primary MMP-3 antibody (SantaCruz sc21732 (1 : 100)) was performed overnight at 4°C. After washing three times, the samples were incubated with a secondary antibody labeled with HRP (GB23303, 1 : 200, Servicebio) for 50 min at room temperature, followed by wash and incubation with the diaminobenzidine substrate (DAKO) for a period controlled under the microscope. Counterstaining was performed with diluted Harris hematoxylin (KIGENE, China). Microscopic results were scanned with the CaseViewer system.

The IHC result was determined by two independent pathologists from Huashan Hospital, Fudan University, Shanghai, China. The pathological section observed a brown-stained area or region for MMP-3 positive granules. Each slice was observed via the CaseViewer system, and the number of positive cells was observed. The MMP-3 expression was graded as negative, weakly positive, medium positive, and strong positive. The point of each grade was: negative (0): lower than 10%; weak positive (1): 11%-40%; medium positive (2): 41%–70%; strong positive (3): higher than 70%.

### 2.15. *In Vivo* Study Assays

10 nude mice (6-8 weeks, male) were randomly divided into 2 groups: 5 in the single gemcitabine (GEM) group and 5 in cordycepin plus gemcitabine (CG) group. The procedure of *in vivo* study is shown in Figure 1(d). In the first, GEM and CG groups were injected with STZ 175 mg/kg after fasting for 12 hours. All mice were injected with 5^∗^10^6^ BxPC-3 pancreatic cancer cells subcutaneously a week later. The fast blood glucose level of the two groups was measured using a glucometer purchased from Yuyue, Shanghai, China. Only when the fasting blood glucose of the mice is over 20 mmolo/L can they be regarded as diabetic mice. Mice in the GEM group were injected abdominally with 50 mg/kg gemcitabine (MCE, Shanghai, China) twice a week. Mice in the CG group were abdominally injected with 50 mg/kg gemcitabine + 30 mg/kg cordycepin twice a week. All animals were sacrificed two weeks after the first injection of drugs. The timeline and schematic diagram of the animal experiment are shown in Figure 1(d).

## 3. Results

### 3.1. Diabetic Status Affects Clinical Outcomes in Pancreatic Cancer Patients

In the TCGA cohort (Figure 2(a)), the diabetic PDA cases had a relatively lower OS level than normal cases in advanced pathological grade patients (median survival: 224 days vs. 652 days, *P* = 0.0075). Similarly, in Figure 2(b), the median overall survival (OS) in the diabetic group and normal group was 501 days and 414 days (*P* = 0.0298) in patients who accepted adjuvant therapy of gemcitabine plus paclitaxel therapy after surgery in Huashan Hospital (Huashan cohort). All patients in the Huashan cohort did not accept neoadjuvant treatment previously. Additionally, in Table 1, diabetic status showed little relationship with gender, age, cancer pathological stages, and metastasis but was positively related to the tumor volume in the Huashan cohort (3.44 cm^3^ vs. 4.407 cm^3^, *P* = 0.003). This result indicated that diabetic patients had a larger tumor volume.

### 3.2. High Glucose Status Promotes Invasion and Gemcitabine Resistance in PDA Cells

We performed laboratory experiments based on the previous clinical findings to ascertain whether high glucose status promotes gemcitabine resistance and cancer invasion *in vitro*. We defined three groups according to different glucose concentrations in cell mediums: 25 mmol/L glucose as the high glucose (HG) group, 15.5 mmol/L as the medium glucose (MG) group, and 5.5 mmol/L as the low glucose (LG) group. We validated the gemcitabine resistance at first. Firstly, after being treated with 10 *μ*mol/L gemcitabine for 24 h, the HG group showed higher cell viability in all pancreatic cancer cell lines than MG and LG (BxPc-3, PANC-1, MiaCaPa-2, PANC-2, and HPDE6-C7) groups (Figure 3(d)). Moreover, after being treated with 10 *μ*mol/L gemcitabine for 24 h, BxPc-3, PANC-1, and MiaCaPa-2 cell lines showed a statistical difference in cell viability between HG, MG, and LG groups in Figure 3(d) (*P* = 0.0069, 0.0386 and 0.0047). Next, HG and MG groups had a higher cell viability rate than the LD group after being treated with gemcitabine for 24 h and 48 h (*P* = 0.0069 and 0.050) (Figure 3(c)). The cancer cell apoptotic rate in HG, MG, and LG after treated with 10 *μ*mol/L gemcitabine for 24 h was 19.8%, 21.9%, and 26.1% (Figure 3(e)). Next, we assessed cancer invasion ability under the gemcitabine environment via the wound healing test. The invasion ability in the HG group was better than the MG group, and the MG group was better than the LG group in the BxPc-3 cell line (Figure 3(f)).

### 3.3. MMP-3 Correlates with Survival and Diabetic Status in PDA

Our clinical and experimental study proved the altered gemcitabine resistance and cancer invasion effect under the high glucose environment. Next, in order to clarify the key factors involved in gemcitabine resistance induced by high glucose status, we applied the RNA sequence data downloaded from the TCGA database. We set two groups: the diabetic group (*n* = 38) and the normal group (*n* = 108), according to the diabetes history in the database. Through differentially expressed gene (DEGs) analysis, 119 genes were differentially expressed within these two groups, shown as the volcano plot in Figure 2(d). And the top 30 differentially expressed genes were presented as a heat map in Figure 2(c). Through pathway enrichment analysis (GO and KEGG analysis), digestive function (pancreatic secretion, fat and protein digestion), serine hydrolase activity, and humoral immune response were enriched signal pathways in the diabetic PDA cohort (Figure 2(f)). Moreover, the GSEA results (Figure 2(e)) showed that diabetic samples were associated with the B cell receptor signal pathway, cell adhesion pathway, chemokine signal pathway, and NADPH oxidase pathway. We then performed a univariate Cox regression analysis and found 19 genes statistically related to the overall survival in PDA patients. We finally used the LASSO regression analysis of these 19 genes and found that MMP-3 had the highest positive coefficient value of 0.11(Figure 3(a)). Based on this, MMP-3 might be an important prognostic factor that participated in the survival reduction of diabetic PDA patients.

We then used clinical resected samples to validate whether MMP-3 was differentially expressed in diabetic PDA samples.  Figure 4(a) showed that in PDA patients, MMP-3 expression was significantly increased in tumor tissue than in the normal pancreatic tissue. IHC test based on surgical samples (Figure 5(a)) showed that MMP-3 expression in protein level was higher in tumor tissue. Compared to euglycemic PDA samples, our result showed diabetic PDA samples had higher MMP-3 expression in both mRNA expression and protein expression levels compared to the normal PDA samples (Figures 4(a) and 5(b)). In Figures 5(b) and 5(c), a significantly higher MMP-3 positive value was found in diabetic PDA samples than the positive value in euglycemic PDA samples (mean positive grade: 2.455 vs. 1.727, *P* = 0.0189). In pancreatic cancer cells, MMP-3 expression was higher in the HG group compared to MG and LG groups. And MMP-3 expression was increased with the elevation of glucose concentration in the medium (Figure 5(d)).

After confirming that MMP-3 was closely related to survival and diabetes in PDA models, we next analyzed the role of MMP-3 in PDA gemcitabine resistance and invasion. Firstly, pan-cancer analysis (Figure 2(g)) revealed that MMP-3, a member of the matrix metalloproteinase family, was overexpressed in many types of solid tumors, including breast cancer (BRCA), cervical cancer (CESC), bile duct cancer (CHOL), colon cancer (COAD), esophageal cancer (ESCA), and pancreatic cancer (PAAD). However, in hematological malignancies, MMP-3 expression was decreased in diffuse large B-cell lymphoma (DLBC) and acute myeloid leukemia (LAML). Next, we set the top 50% MMP-3 expression level in the TCGA-PAAD cohort as the high MMP-3 group and the rest as the low MMP-3 group. In the TCGA database (Figure 4(b)), reduced survival was found in the high MMP-3 group in the whole PDA patients (median survival: 532 days vs.702 days, *P* = 0.001) and gemcitabine users (median survival: 394days vs. 691days, *P* = 0.019). The MMP-3 prognostic prediction efficacy was performed by ROC curve analysis. The area under the curve (AUC) of 1-year, 3-year, and 5-year survival was 0.604, 0.655, and 0.712 (Figure 4(c)).  Table 2 was the clinical baseline information in MMP-3 differently expressed groups. MMP-3 was positively related to histological grade (*P* = 0.008) and overall survival (*P* < 0.001). Through DEGs analysis, GO analysis (Figure 4(f)), and GSEA analysis (Figures 4(d) and 4(e)), we found neuronal system, transmission across chemical synapses, drug metabolism, degradation of the extracellular matrix, extracellular matrix organization, matrix metalloprotease, and oxidative stress-related pathways were enriched in the higher MMP-3 expressed group.

### 3.4. MMP-3 Is Related to Gemcitabine Resistance and Cancer Invasion

We performed a series of laboratory studies to validate the function of MMP-3 in PDA gemcitabine resistance and invasion. We used two MMP-3 siRNAs (MMP-3_Si01 and MMP-3_Si02) and cordycepin, a selective MMP-3 inhibitor, to test the effect of blocking MMP-3 in pancreatic cancer cells. In Figures 5(e) and 5(f), siRNAs (MMP-3_Si01, MMP-3_Si02) and cordycepin significantly inhibited MMP-3 expression compared with normal control (NC_1). And the apoptosis of BxPc-3 cells was higher in MMP-3 siRNAs (MMP-3_Si01, MMP-3_Si02) and 20 *μ*mol/L cordycepin treated groups compared with normal control (NC_1) (Figures 5(g) and 5(h)) under 10 *μ*mol/L gemcitabine environment. Meanwhile, overexpressing MMP-3 (MMP-3_OVER) elevated BxPc-3 cell survival and reduced apoptosis in the 10 *μ*mol/L gemcitabine environment (Figures 5(g) and 5(h)). Compared with normal control, cancer invasion was increased in the MMP-3_OVER group and decreased in the siRNA (MMP-3_Si01) treated group compared with normal control (*P* < 0.001) (Figure 6(a)). In the normal control group, 10 mmol/L cordycepin+10 *μ*mol/L gemcitabine and 20 mmol/L cordycepin+10 *μ*mol/L gemcitabine treated group, the cell viability of pancreatic cancer cells decreased with higher cordycepin concentration (Figure 6(g)). What is more, in Figure 1(b), the difference in cell viability between HG, MG, and LG was also decreased in the 20 mmol/L cordycepin+10 *μ*mol/L gemcitabine treated group than the 10 mmol/L cordycepin+10 *μ*mol/L gemcitabine treated group.

Next, we measured the effect of blocking MMP-3 in the naturally generated gemcitabine-resistant cell line. The MMP-3 expression was elevated in naturally generated gemcitabine-resistant cancer cells than in normal cancer cells (Figure 1(c)). Under single 10 *μ*mol/L gemcitabine treatment, gemcitabine resistant cell line (BxPc-3 (GemR)) showed higher cell viability (0.955 vs. 0.787, *P* = 0.0026) than the normal cell line (BxPc-3 Normal) (Figure 1(e)). However, compared with the single gemcitabine treated group, gemcitabine plus cordycepin and gemcitabine plus setanaxib effectively reduced cell viability (Figure 1(e)). In Figure 1(e), gemcitabine resistant cell line showed a statistically higher cell viability rate than the normal group in the cordycepin plus gemcitabine group (0.7068 vs. 0.6438, *P* = 0.0104) and the setanaxib group (0.8545 vs. 0.7498, *P* = 0.0107). But the difference value between BxPc-3 (GemR) and BxPc-3 (Normal) was reduced in the gemcitabine plus cordycepin treatment group than in the single gemcitabine treated group (0.063 vs. 0.168). In comparison, the difference value was larger in the setanaxib plus gemcitabine group (0.105 vs. 0.168).

Finally, we confirmed our findings *in vivo* using a diabetic pancreatic cancer mouse model. The schematic diagram of the *in vivo* study is shown in Figure 1(d). After constructing the diabetes model, 10 nude mice (6-7 weeks) were randomly divided into 2 groups: GEM (50 mg/kg) group and cordycepin (30 mg/kg) plus GEM (50 mg/kg) (CG) group. The survival plot of these two groups is shown in Figure 1(f). Two mice died on day 20 and day 25 in the GEM group, and two died on day 14 and day 27 in the GEM plus 30 mg/kg cordycepin (CG) group (*P* = 0.9873). The result of tumor volume was 0.8357 ± 0.2483 cm^3^ in the GEM group and 0.4093 ± 0.0547 cm^3^ in the CG group (*P* = 0.0445) (Figure 1(h)). Obviously, the CG group showed smaller tumor volume and death rate after accepting drug injections.

### 3.5. Gemcitabine Metabolism-Related Gene RRM1 Is Associated with MMP-3 Expression

Previous studies demonstrated that nucleoside transporters (NTs) family (ENT1 (SLC29A1), CNT1 (SLC28A1), CNT3 (SLC28A3)), ribonucleotide reductase (RR) family (RRM1, RRM2), excision repair cross-complementation 1 (ERCC1), PLK1, and multiple-drug resistant protein 1 (MRP1, ABCB1) were vital in the metabolic process of gemcitabine in pancreatic cancer cells [3]. In the TCGA database, MMP-3 showed a statistical relationship with CNT1, CNT3, RRM1, and RRM2 (*P* < 0.05) in Figure 4(f).  Figure 4(h) demonstrated that MMP-3 showed a relatively weaker positive relationship with CNT1 and CNT3, while MMP-3 revealed a stronger relationship with RRM1 and RRM2. We then found that only RRM1 expression (1.156 vs. 0.85, *P* = 0.0285) was significantly increased in the 100 U MMP-3 treated pancreatic cells than the normal control according to the data from GSE50931. Moreover, RRM2 (1.192 vs. 0.879, *P* = 0.1415), CNT1 (0.988 vs. 0.976, *P* = 0.4332), and CNT3 (0.954 vs. 1.009, *P* = 0.8548) expressions showed no statistical difference under the stimulation of 100 U MMP-3 than the normal control group. The results are shown as the heat map in Figure 4(i).

### 3.6. ROS Is Involved in High Glucose-Induced MMP-3 Overexpression

Next, we tested whether ROS was involved in the mediation of MMP-3. It is generally accepted that high glucose stimulates reactive oxygen species (ROS) to alter a series of cell metabolism. From bioinformatical results, the NADPH oxidase pathway (Figure 2(e)) was enriched in the diabetic cohort, and the oxidative stress (Figure 4(e)) was enriched in the high MMP-3 expression cohort. In Figure 3(b), ROS level was also increased in HG and MG compared to LG (*P* < 0.001). And in Figure 5(d), NOX4 expression was increased with the elevation of glucose concentration.  Figure 4(g) revealed that MMP-3 expression was strongly associated with NOX4 rather than NOX1 in pancreatic cancer. And in Figure 6(b), NOX4 showed a positive relationship with NOX in TCGA pancreatic cancer cohort (*r* = 0.391, *P* < 0.001). Taken together, it was logical to suppose that ROS mediated by NOX4 might participate in MMP-3 overexpression regulated by high glucose.

We then performed experiments to prove the role of NOX4-mediated ROS in MMP-3 overexpression. Firstly, in Figure 6(d), the setanaxib, a selective NOX4 inhibitor, effectively suppressed both NOX4 and MMP-3 expression compared to the normal control group in cancer cells. However, in H_2_O_2_, a potent ROS stimulator, treated group, MMP-3, and NOX4 expression were both increased compared to the normal control. But MMP-3 siRNAs treated groups and the cordycepin treated group did not show an apparent change in NOX4 expression (Figure 5(e)). And MMP-3 overexpression group did not affect the NOX4 expression level (Figure 5(e)). This result indicated that ROS might be an upstream factor in the MMP-3 activation. Moreover, the NOX4 expression in pancreatic cancer cells did not showed an obvious change after being treated with 100 U MMP-3 in the GSE50931 (Figure 4(i)). Finally, after treated with 20 *μ*mol/L setanaxib for 24 h, the MMP-3 and NOX4 expression were similar between the HG, MG, and LG groups compared with the normal group (Figures 6(c) and 6(d)).

### 3.7. ROS Participates in High Glucose-Induced GEM Resistance and Invasion

We finally confirmed whether ROS was an intermediate factor involved in the gemcitabine resistance and cancer invasion caused by high glucose. Firstly, we observed increased ROS levels in HG and MG compared to LG (0.8855, 0.8115, 0.7910, *P* < 0.001) (Figure 3(b)). In Figure 6(d), H_2_O_2_ increased NOX4 expression and setanaxib decreased NOX4 expression in BxPc-3 cell lines.  Figure 6(f) demonstrated that HG, MG, and LG groups showed increased cell viability after treated with 50 *μ*mol/L and 10 *μ*mol/L H_2_O_2_ for 24 h compared with the single GEM treated group. Using setanaxib plus GEM, the cell viability was reduced in HG, MG, and LG groups (Figures 1(b) and 6(f)). The cell viability was also decreased with the decrease of H_2_O_2_ concentration and the increase of setanaxib concentration (Figure 6(f)). The difference between HG, MG, and LG was decreased with the increase with the elevation of H_2_O_2_ concentration and the senataxib concentration. Secondly, targeting NOX4 mediated ROS also influenced PDA invasion under the gemcitabine environment. In Figure 6(e), BxPc-3 cells treated with 10 *μ*mol/L H_2_O_2_+10 *μ*mol/L GEM, 20 *μ*mol/L setanaxib+10 *μ*mol/L GEM, and single 10 *μ*mol/L GEM showed statistical difference in Transwell study. Interestingly, in Figure 1(a), the tumor-suppressive effect of single cordycepin was similar to the effect of single setanaxib treatment. But in Figure 1(b), 20 *μ*mol/L cordycepin+10 *μ*mol/L gemcitabine group showed better tumor-suppressive effect than 20 *μ*mol/L setanaxib+10 *μ*mol/L gemcitabine. Based on this, the MMP-3 inhibitor may be a better gemcitabine sensitizer compared to the NOX4 inhibitor.

## 4. Discussion

With the elevation of life quality, it is foreseeable that the incidence of diabetes will continue to rise for a long time in the future. Diabetes mellitus was a signal of poor prognosis found in many studies from American and Asian gemcitabine users [6–10]. Our study elucidated that DM might lead to a worse clinical outcome in Chinese PDA patients. As the main characteristics of diabetes, increased blood glucose level is essential for pancreatic cancer development and resistance to therapies. High glucose cannot only work as a direct energy supply for cancer cells to grow much faster but also stimulate multiple signal pathways, which are essential for pancreatic cancer development [11]. Our study provides a novel insight into that high glucose may directly strengthen gemcitabine resistance and invasion via ROS/MMP-3 signaling pathway.

At first, we confirmed the association between gemcitabine resistance with glucose concentration from clinical data and laboratory experiments. Our clinical retrospective result demonstrated that diabetes signals poor clinical outcomes in PDA patients, especially in PDA gemcitabine users. Gemcitabine is the first-line chemical drug in PDA treatment. Gemcitabine mainly interferes with DNA synthesis to induce apoptosis in pancreatic cancer cells to inhibit cancer progression. So, we tested the cell viability, apoptosis, and wound-healing rate to measure the gemcitabine sensitivity and cancer invasion in pancreatic cancer cells under different glucose concentrations. Then, through survival-related univariate study and LASSO regression analysis, we focused our interest on MMP-3, a matrix metalloprotease. And we also found that MMP-3 expression was correlated with high glucose status in PDA through clinical samples, bioinformatical sequencing, and laboratory experiments.

From clinical samples, bioinformatical results and cellular experiments, we found that MMP-3 expression was related to high glucose status in pancreatic cancer. MMP-3, a member of the matrix metalloproteinase family, is well-known as a vital factor in cancer metastasis and invasion. MMP-3 promotes cancer invasion and metastasis through the enzymic breakdown of the basal membrane and extracellular matrix. Our study found that MMP-3 expression was upregulated in many solid malignant tumors. In pancreatic cancer, MMP-3 was reported to be related to cancer invasion and metastasis [12]. This might be the reason why we observed increased PDA invasion under a higher glucose environment. Our study also confirmed that inhibiting MMP-3 expression significantly reduced PDA invasion under the gemcitabine environment. Moreover, MMPs have also been reported to alter cancer cell proliferation and antiapoptosis through the crosstalk with multiple signal pathways. Our result showed that MMP-3 effectively blunted PDA gemcitabine sensitivity, which presented as reduced apoptosis and promoted proliferation in pancreatic cancer cells. During this process, we furtherly found that cordycepin, a selective MMP-3 inhibitor, had a satisfying effect in suppressing pancreatic cancer gemcitabine resistance. Cordycepin is a derivative from the fungal genus *Cordyceps militaris* and has long been used as an active pharmacological ingredient in traditional Chinese medicine. Cordycepin was reported to inhibit MMP-3 expression in many inflammatory diseases [13–16]. In the *in vivo* study, the GEM+cordycepin group showed a reduced tumor volume than the single gemcitabine treated group. Additionally, MMP-3 was also reported to be closely related to diabetic inflammatory complications. Blocking MMP-3 expression significantly decreased the rate of diabetes-related complications in many animal models. Our study found that diabetic PDA cases were closely related to inflammation. After accepting chemotherapy, reduced mortality in the GEM+cordycepin group indicated that blocking MMP-3 can suppress gemcitabine resistance and increase mice's tolerance to drugs in DM animal models. MMP-3 may be a potential novel target for suppressing gemcitabine resistance and reducing diabetic complications simultaneously, which may benefit many diabetic PDA victims.

Additionally, we explored the potential downstream signal effectors of MMP-3 in gemcitabine resistance because MMP-3 did not directly participate in gemcitabine metabolism in PDA. CNT1, CNT3, RRM1, and RRM2 were statistically positively related to MMP-3 expression. These four genes were reported to influence gemcitabine metabolism in PDA directly. CNT1 and CNT3 worked as transporter to carry gemcitabine into the cell nucleus. Because of this, increased CNT1 and CNT3 could lead to elevated gemcitabine sensitivity [17, 18]. Reversely, RRM1 and RRM2 were associated with the repairment of DNA structure which is essential for countering the DNA damage effect by gemcitabine. Moreover, data from the GEO database furtherly supported that only RRM1 expression is statistically upregulated by MMP-3 stimulation. RRM1 was found to be upregulated in gemcitabine-resistant pancreatic cancer cells [19]. And it was also reported as an independent prognostic factor in pancreatic cancer patients [20]. RRM1 was reported to accumulate at the DNA damage sites and facilitate damage repairment which helps pancreatic cancer cells to overcome the apoptosis induced by gemcitabine. The silence of RRM1 effectively increased gemcitabine accumulation by enhancing the expression of uptake transporters. Unfortunately, the regulation of RRM1 in pancreatic cancer is still not clear. At present, only the RAS/ERK signaling pathway was reported to regulate the expression of RRM1 [21]. Because of this, it is not clear whether MMP-3 directly promotes RRM1 or indirectly promotes RRM1 expression via signal pathways such as the RAS/ERK signaling pathway. More study on the interaction between RRM1 and MMP-3 in pancreatic cancer is urgently needed in the future.

We also noticed ROS might be an intermediate factor in the high glucose-mediated MMP-3 overexpression. Previous studies found that MMP-3 was regulated by ROS in many models, including pancreatic cancer cell model [22]. Our GSEA result observed an enriched NADPH oxidase pathway in the DM group. The enriched oxidative stress was found in the high MMP-3 expressed group, which indicated NADPH oxidase and ROS might participate MMP-3 related signal pathways. ROS, a group of oxygen-containing chemicals, is an important regulator in many signal pathways. For cancer cells, ROS is essential for tumorigenesis and oncogene initiation. ROS stimulates antioxidation signal pathways to enhance the survival and proliferation of cancer [23].In PDA, ROS level is mainly regulated by NADPH oxidase 4 (NOX4) [24]. The NOX4 expression level directly reflects the ROS level in pancreatic cancer cells and in our study, both elevated ROS and NOX4 expression were found in higher glucose concentration groups [25]. Taken together, it is logical to suppose that MMP-3 may be regulated by ROS, which is initiated by high glucose.

This hypothesis that NOX4-related ROS mediated MMP-3 expression is then validated in our study. Our result indicated that ROS might be the bridge that links a high glucose environment with MMP-3 overexpression. Our *in vitro* study found stimulating NOX4 expression via H_2_O_2_ or blocking NOX4 expression via setanaxib significantly influenced MMP-3 expression. Setanaxib, a selective NOX4 inhibitor, is a critical ROS inhibitor undergoing clinical trials for cancer therapies, while H_2_O_2_ was a strong ROS promoter in cancer cells [26, 27]. Through using setanaxib, the MMP-3 expression was similar in HG, MG, and LG. Reversely, interfering MMP-3 expression could not influence NOX4 expression. Single MMP-3 stimulation showed little influence on NOX4 expression from our experimental result and the bioinformatical analysis of GSE50931. As a result, ROS mediated by NOX4 is the upstream signal factor of MMP-3. We also found ROS mediates gemcitabine resistance and cancer invasion altered by a high glucose environment. Blocking NOX4 expression effectively inhibited PDA invasion and gemcitabine sensitivity. And the difference in cell viability between HG, MG, and LG was also reduced when treated with setanaxib. Because of this, ROS may be the intermediate factor in the mechanism of gemcitabine resistance caused by high glucose.

Interestingly, blocking MMP-3 had a better tumor-suppressive effect in gemcitabine-treated pancreatic cancer cells than blocking ROS. And we also found the gemcitabine resistance of the high glucose group was most elevated in 10 *μ*mol/L H_2_O_2_ treated HG group, not the 50 *μ*mol/L H_2_O_2_ treated group. This may be because ROS is a double-edged sword in PDA development. ROS promotes cancer progression and induces chemoresistance to protect cancer cells from apoptosis within certain limits. However, exposure to an extremely high ROS level will directly cause DNA damage in cancer cells, thus leading to apoptosis. Based on this, ROS inhibition could lead to a dual inhibition in tumor apoptosis and antiapoptosis [28]. Moreover, ROS was reported to be generated by gemcitabine to impair DNA structure in pancreatic cancer. And this elevated ROS induced by gemcitabine may explain why MMP-3 was overexpressed in the naturally generated gemcitabine-resistant pancreatic cancer cells from another aspect.

## 5. Conclusion

In this project, we discovered that diabetic status or a high-glucose environment played as a vital role in PDA gemcitabine resistance and invasion, which significantly reduced the survival of pancreatic cancer patients. High glucose elevates gemcitabine resistance via upregulating ROS levels to stimulate MMP-3 overexpression in pancreatic cancer cells. *In vivo* and *in vitro* experiments revealed that targeting MMP-3 effectively relieved gemcitabine resistance and suppressing MMP-3 expression showed a batter effect than inhibiting ROS level. And RRM1 may be the potential downstream factor activated by MMP-3 in the high glucose-mediated gemcitabine resistant metabolism.

## Figures and Tables

**Figure 1:** (a) Different glucose groups (HG, MG, and LG) BxPc-3 cells treated with normal control (NC), single 10 *μ*mol/L GEM group, single 20 *μ*mol/L setanaxib, and single 20 *μ*mol/L cordycepin. (b) Different glucose groups (HG, MG, and LG) BxPc-3 cells treated with single 10 *μ*mol/L GEM group, 10 *μ*mol/L setanaxib+10 *μ*mol/L GEM group, and 20 *μ*mol/L setanaxib+10 *μ*mol/L GEM group, 10 *μ*mol/L cordycepin+10 *μ*mol/L GEM group, and 20 *μ*mol/L cordycepin+10 *μ*mol/L GEM group. (c) MMP-3 expression in natural generated gemcitabine resistant cell line (BxPc-3 (GemR)) and in normal control (BxPc-3 (Normal)). (d) The schematic diagram and the timeline of the *in vivo* experiment in nude mouse. (e) The cell viability of BxPc-3 (GemR) and BxPc-3 (Normal) after treated with10 *μ*mol/L GEM, 20 *μ*mol/L setanaxib+10 *μ*mol/L GEM, and 20 *μ*mol/L cordycepin+10 *μ*mol/L GEM for 24 h. (f) The K-M survival plot of the mice in the GEM+cordycepin treated group, and single GEM treated group (*P* = 0.9875). (g, h) Tumor volume comparison between GEM + cordycepin treated diabetic group and single GEM treated group (^∗^*P* < 0.05).

**Figure 2:** (a, b) K-M survival plots of PDA patients in TCGA cohort (A) and PDA gemcitabine users in Huashan cohort (B). (c) Heat map of the top 30 genes differentially expressed between the normal and the diabetic PDA patients (blue = normal group, red = DM group). (d) Volcano plot of DEGs between normal and diabetic PDA patients in TCGA database (up: upregulated genes, down: downregulated genes). (e) GSEA analysis of pathways enriched in the diabetic group. (f) GO and KEGG analyses of the pathways enriched in the DM group. (g) Pan-cancer analysis of MMP-3 expression between the normal tissue and the cancerous tissue based on the TCGA database (^∗^*P* < 0.05, ^∗∗^*P* < 0.01, ^∗∗∗^*P* < 0.001).

**Figure 3:** (a) Lasso regression analysis of DEGs between the normal and the DM groups. (b) ROS level of BxPC-3 cell lines under different glucose levels (HG: high glucose level group, MG: medium glucose level group, LG: low glucose level group). (c) Cell viability of BxPc-3 treated with 10 *μ*mol/L gemcitabine for 24 h and 48 h. (d) Pancreatic cancer cell lines were treated with 10 *μ*mol/L gemcitabine for 24 h under different glucose levels. (e) The apoptosis rate of different glucose groups under 10 *μ*mol/L gemcitabine for 24 h (the lower right is the bar graph concluding the apoptosis between three groups). (f) Wound healing test of different glucose levels.

**Figure 4:** (a) Left: MMP-3 expression between normal tissue and the PDA tissue; Right: MMP-3 expression between normal PDA patients and the person with diabetes (DM) PDA patients (^∗^*P* < 0.05, ^∗∗∗^*P* < 0.001). (b) ROC curve of MMP-3 predicting the overall survival of PDA patients in 1-year, 3-years, and 5-years. AUC (area under the curve) measures the predicting efficacy of MMP-3 in different time models. (c) K-M survival plot of the high MMP-3 group, and the low MMP-3 group in the TCGA pancreatic cancer cohort (left) and TCGA PDA gemcitabine users (right). (d, e) GSEA analysis of pathways enriched in high MMP-3 group. (f) GO and KEGG analyses of the pathways enriched in high MMP-3 group. (g, h) Heat map of the association between the single genes (ENT1 (SLC29A1), ENT3 (SLC29A3), CNT1 (SLC28A1), CNT3 (SLC28A3), RRM1, RRM2, MRP1 (ABCB1), NOX1, NOX4, and PLK1) expression and the MMP-3 expression in PDA cohort (^∗^*P* < 0.05, ^∗∗∗^*P* < 0.001). (i) The expression of NOX4, RRM1, RRM2, CNT1, and CNT3 in 100 U MMP-3 treated pancreatic cancer cell line and normal control group from GSE50931 (ns: not significant (*P* > 0.05), ^∗^*P* < 0.05).

**Figure 5:** (a) MMP-3 expression in normal pancreas tissue (left) and in PDA tissue (right) (downloaded from https://www.proteinatlas.org). (b, c) MMP-3 expression difference between normal (*n* = 11) (left) and diabetic PDA patients (*n* = 11) (right) (^∗^*P* = 0.0198). (d) MMP-3 expression in high, medium, and low glucose group (e) MMP-3, beta-actin, and NOX4 expression in MMP-3 siRNAs treated group (MMP-3_Si01 and MMP-3_Si02), 20 *μ*mol/L cordycepin, MMP-3 overexpression group (MMP-3_OVER), and normal control (NC_1) (^∗∗∗^*P* < 0.001, ns:>0.05). (f) The grey value of MMP-3/beta-actin and NOX4/beta-actin in Figure 1(e). (g) Apoptosis analysis of MMP-3 siRNAs treated group (MMP-3_Si01 and MMP-3_Si02), 20 *μ*mol/L cordycepin, MMP-3 overexpression group (MMP-3_OVER), and normal control (NC_1 and NC_2). (h) The bar plot of the apoptotic rate in MMP-3_OVER, NC_1, NC_2, MMP-3_Si01 MMP-3_Si02, and 20 *μ*mol/L cordycepin treated group.

**Figure 6:** (a) Transwell analysis of MMP-3 overexpression group (MMP-3_OVER), normal control (NC_1), and MMP-3 silencing group (MMP-3_Si01) (^∗∗∗^*P* < 0.001) under 10 *μ*mol/L gemcitabine environment. (b) Spearman analysis of the association between NOX4 and MMP-3 in TCGA database. (c) NOX4 and MMP-3 expression in 20 *μ*mol/L setanaxib treated high glucose, medium glucose, and low glucose group. (d) MMP-3 and NOX4 expression in 10 *μ*mol/L H_2_O_2_ group, 20 *μ*mol/L NOX inhibitor (setanaxib), 10 *μ*mol/L NOX inhibitor (setanaxib), 10 *μ*mol/L cordycepin, and normal control (NC_1). (e) Transwell analysis of 10 *μ*mol/L H_2_O_2_ group, normal control (NC_1), and 20 *μ*mol/L NOX inhibitor (setanaxib). (f) The cell viability of BxPc-3 cells treated with 50 *μ*mol/L H_2_O_2_+10 *μ*mol/L gemcitabine (GEM) group, 10 *μ*mol/L H_2_O_2_+10 *μ*mol/L GEM group, single 10 *μ*mol/L GEM group, 5 *μ*mol/L setanaxib+10 *μ*mol/L GEM group, 10 *μ*mol/L setanaxib+10 *μ*mol/L GEM group, and 20 *μ*mol/L setanaxib+10 *μ*mol/L GEM group under different glucose groups (HG, MG, and LG). (g) The cell viability of BxPc-3 cells treated with 10 *μ*mol/L GEM group, 10 *μ*mol/L GEM+10 *μ*mol/L cordycepin group, and 10 *μ*mol/L GEM+20 *μ*mol/L cordycepin group under different glucose groups (HG, MG, and LG).

**Table 1:** The baseline information of PDA patients (*n* = 129) from Huashan Hospital.

Characteristics	Normal	DM	*P* value
Overall cases	87	42	
Age	62.91 (39-86)	63.69 (50-77)	0.59
Sex (male)	54	22	0.295
Pathological stage			0.613
I-II	56	22	
III-IV	31	20	
Metastasis	8	6	0.384
Tumour volume	3.44 (0.80-12)	4.407 (1.6-10)	**0.003**

**Table 2:** Baseline information of MMP-3 differently expressed groups (TCGA database).

Characteristic	MMP3(low)	MMP3(high)	*P* value
Overall cases	89	89	
T stage, *n* (%)			0.290
T1	4 (2.3%)	3 (1.7%)	
T2	16 (9.1%)	8 (4.5%)	
T3	66 (37.5%)	76 (43.2%)	
T4	1 (0.6%)	2 (1.1%)	
*N* stage, *n* (%)			0.375
N0	28 (16.2%)	22 (12.7%)	
N1	58 (33.5%)	65 (37.6%)	
*M* stage, *n* (%)			0.672
M0	38 (45.2%)	41 (48.8%)	
M1	3 (3.6%)	2 (2.4%)	
Pathologic stage, *n* (%)			1.000
I-II	83 (47.4%)	84 (48%)	
III-IV	4 (2.3%)	4 (2.2%)	
Sex (male)	53 (29.8%)	45 (25.3%)	0.292
Histologic grade, *n* (%)			**0.008**
G1	23 (13.1%)	8 (4.5%)	
G2	39 (22.2%)	56 (31.8%)	
G3	25 (14.2%)	23 (13.1%)	
G4	1 (0.6%)	1 (0.6%)	
OS event, *n* (%)			**<0.001**
Alive	55 (30.9%)	31 (17.4%)	
Dead	34 (19.1%)	58 (32.6%)	
Age	67 (58-73)	65 (57-73)	0.448

## Data Availability

The RNA sequence data can be downloaded from https://portal.gdc.cancer.gov (The TCGA-PAAD cohort).
